The article "Econometric Analysis of Leisure Agriculture and Rural Tourism Scenery Based on Spatial Data Analysis" was retracted in 2023. Reasons: unreliable results or conclusions; concerns about the data; concerns about the peer review; concerns about the citations.

# Econometric Analysis of Leisure Agriculture and Rural Tourism Scenery Based on Spatial Data Analysis

**DOI:** 10.1155/2022/2286803

**Published:** 2022-07-18

**Authors:** Shihui Liu, Bing Gao

**Affiliations:** ^1^Guangzhou College of Commerce, Guangzhou, Guangdong 511363, China; ^2^Chinese Academy of Natural Resources Economics, Xicheng, Beijing 100035, China

## Abstract

Exploratory spatial data analysis (ESDA) shows that there is a significant spatial autocorrelation of tourism development in China, which is manifested by the aggregation of spatial distribution. The results of the great likelihood estimation of the spatial lag model show that the parameters *ρ* of both the total tourism income model and the domestic income model are significantly positive, indicating that the spatial linkage between agricultural and rural tourism income is very strong and the spillover effect of agricultural and rural tourism is larger than that of overall tourism. Tourism superstructure facilities, human resources, and tourism infrastructure are statistically significant and are important influencing factors for overall tourism and agricultural and rural tourism development. And the overall fit of agricultural and rural tourism model is poor. The findings of the study better grasp how to make rural tourism make a greater contribution to the regional economy of Chengdu and maximize its positive role, and put forward relevant countermeasure suggestions, which will provide theoretical guidance and decision-making reference for relevant departments on how to better play the economic effect of tourism, and will also have a realistic reference role on how to develop rural tourism in western cities of China.

## 1. Introduction

Agriculture is a vibrant and priority industry in China, and as a large agricultural country, agricultural economic growth is an important issue in China. Since the end of the 20th century, agricultural productivity has been liberated with the introduction of a series of policies to support and benefit agriculture [1]. At present, China vigorously implements the strategy of rural revitalization, allowing the integrated development of rural one, two, and three industries, so as to promote farmers' income, rural prosperity, and agricultural efficiency, and industrial integration development is the only way to revitalize the countryside [2]. The 2019 Central Government Document No. 1 proposes to make use of rural special industries and cultural connotations, develop leisure tourism and catering B&B that can meet the needs of urban and rural residents, realize the optimal allocation of rural resources, and develop new service industry in the countryside. The integration of agriculture with other industries, especially with tourism, is becoming a new driving force for agricultural economic growth, and rural tourism has become an effective way to promote the re-employment of farmers and improve the rural environment [3].

The article "Econometric Analysis of Leisure Agriculture and Rural Tourism Scenery Based on Spatial Data Analysis" was retracted in 2023. Reasons: unreliable results or conclusions; concerns about the data; concerns about the peer review; concerns about the citations.

Nowadays, the development scale of China's tourism industry has ranked among the top in the world, maintaining a steady and rapid growth overall, with domestic tourist reception reaching 5.54 billion in 2018, an increase of 10.8% over the previous year, and agricultural and rural tourism income reaching 512.78 billion yuan. The traditional tourism development model has allowed a large number of natural resources to be consumed or even destroyed, while the diversification and personalization of tourism products are increasingly valued by tourists as they increasingly demand material culture [4]. The constraints of income, time, and lagging paid leave system have prompted suburban and weekend trips to be favored by more and more travelers as the preferred way to carry out parent-child activities and leisure and entertainment.

Rural tourism has a positive impact on regional economic income and employment. By comparing current scholarly research on the connotations of rural tourism and economic growth, it is clear that most studies have addressed the micro aspects, while fewer studies have explored the macro aspects of the impact on regional economies [5]. In terms of the methodology of rural tourism research, mainly qualitative research, mostly case studies, empirical research, and tourism planning, has not yet formed a systematic methodology, and the research and development of rural tourism is extremely exploratory [6]. In this paper, we take the life cycle effect theory, economic growth theory, multiplier theory, and the development of rural tourism. Based on economic growth theory, multiplier theory, and tourism economic effect theory, this paper studies the impact of rural tourism on the regional economy of Chengdu, which adds to a certain extent to the research method of rural tourism and enriches the research theory in this field with theoretical reference significance.

The purpose of this paper is to study the impact of agricultural and rural tourism on the regional economy, and it is known that the income from rural tourism will lead to economic growth, what will be the impact on other aspects of the regional economy, how much does rural tourism revenue and income from rural tourism contribute to regional GDP? By using empirical analysis based on current research on agricultural and rural tourism and related industries, this paper explores the income effects of rural tourism on the regional economy, using qualitative analysis to study the employment effects and investment effects of rural tourism [7]. The conclusions of the study better grasp how to make rural tourism make a greater contribution to the regional economy of Chengdu, maximize the positive effects, and put forward relevant countermeasure suggestions, which will provide theoretical guidance and decision-making reference for the relevant departments on how to better play the economic effects of tourism, and will also have some realistic reference role on how to develop rural tourism in western cities of China [8].

The article "Econometric Analysis of Leisure Agriculture and Rural Tourism Scenery Based on Spatial Data Analysis" was retracted in 2023. Reasons: unreliable results or conclusions; concerns about the data; concerns about the peer review; concerns about the citations.

## 2. Related Work

Through combing the literature, it is found that the current research on rural tourism mainly focuses on the concept, development model, type of operation, market and product, and impact.

Regarding the typology of rural tourism, the study [9] argues that functionally, rural tourism can be divided into tasting, farming, healing, ornamental, vacation, and entertainment types; structurally, tourism agriculture can be divided into tourism agriculture, forestry, animal husbandry, and fishery, tourism plantation, and tourism sideline. The authors in [10] divided tourism in terms of function, and they believed that it could be divided into leisure type, sightseeing type, science popularization type, and cultural type. The study [11] has a different opinion; she believes that rural tourism can be divided into folklore, leisure, and sightseeing types in terms of purpose. The author in [12] believes that rural tourism can be divided from several aspects such as geographic location, objects, resources, and scientific content. Geographically, there are scenic area-dependent, suburban, and fringe types.

Regarding the impact of rural tourism, this aspect mainly focuses on the study of the three influencing factors of economy, culture, and environment. According to Zhang Xiang-rang, the rural tourism developed in the glass village of Pinggu District, Beijing, has had a positive effect on the local culture, economy, and management. The authors in [13] selected different research perspectives and used a combination of qualitative and quantitative analysis methods to study in depth the relationship between cultural heritage and rural tourism from the perspectives of villagers, tourists, and researchers, respectively, and concluded that rural tourism can contribute to cultural heritage. The authors in [14] researched the Three Gorges Chexi Folklore Scenic Area in the field and analyzed the influence of local residents on rural tourism using resident perception theory. The authors in [15] took another approach to change the perspective, and they chose rural women as the research object and studied the relationship between women and rural tourism in a village in Lin'an City. The authors in [16] concluded that rural tourism can transfer surplus labor, improve farmers' income, and promote the development of agriculture and related industries. In terms of social and humanistic impacts, the role of rural tourism focuses on the impact of rural culture by strong urban culture, including positive and negative impacts on the environment.

The article "Econometric Analysis of Leisure Agriculture and Rural Tourism Scenery Based on Spatial Data Analysis" was retracted in 2023. Reasons: unreliable results or conclusions; concerns about the data; concerns about the peer review; concerns about the citations.

In terms of the problems and countermeasure suggestions for rural tourism, the author in [17] argues that the current domestic rural tourism mainly has the problems of insufficient rural tourism development characteristics, service management still needs to be standardized, supporting facilities are not sound enough, and tourism product marketing lacks novelty and puts forward countermeasure suggestions on these aspects. The authors in [18] argued that the current development problems of rural tourism are mainly reflected in the dominance of small-scale business entities with family units, thus rural tourism products are too lacking in traditional cultural flavor also too single, basically food-oriented, and the division of labor is not clear enough, and they believe that rural tourism should maintain the local cultural flavor. The authors in [19], in the study of the impact of rural tourism on poverty alleviation, also concluded the current problem of rural tourism products without regional characteristics, if the inclusion of experiential products will be able to increase the competitiveness of rural tourism. The authors in [20] used the classical SWOT analysis to conduct an in-depth analysis of the strengths, weaknesses, opportunities, and threats of urban agriculture in Chengdu, analyzed the current situation, characteristics, and problems including urban agriculture in Chengdu, and conducted an empirical study of urban agriculture models and proposed corresponding countermeasures for the mentioned models, for example, popularizing knowledge and changing citizens' concepts about developing and developing rural tourism products; innovating the investment and financing mechanism of rural agriculture; optimizing the regional layout of urban agriculture; and improving the land transfer system.

## 3. Concept Identification

### 3.1. The Concept of Leisure Agriculture

With the vigorous development of leisure agriculture, the theories about leisure agriculture are also increasing, and many domestic scholars have conducted in-depth research on its theory and practice and have also produced some views. Taiwan was the first region to develop leisure agriculture and has achieved some success, so the term leisure agriculture comes from Taiwan in China. Therefore, the term Leisure agricultural was introduced from Taiwan in mainland China, but after its introduction, there are various translations, such as tourism agriculture and tourism agriculture. Some scholars believe that the term “leisure agriculture” should be standardized to replace “tourism agriculture.”

The article "Econometric Analysis of Leisure Agriculture and Rural Tourism Scenery Based on Spatial Data Analysis" was retracted in 2023. Reasons: unreliable results or conclusions; concerns about the data; concerns about the peer review; concerns about the citations.

### 3.2. The Relationship between Rural Tourism and Leisure Agriculture

Hoyland and Murphy argue that both rural tourism (farm tourism) and leisure agriculture are related to direct agriculture. These two concepts are often interchangeable. However, the difference between the two is defined in two main ways. Farm tourism refers to a tourist's brief stay on a farm, or recreational and leisure activities directly or indirectly on a farm. Agrotourism, on the other hand, refers to residing in an agriculture-related environment that can gradually replace traditional agricultural production functions as tourism activities are carried out, as the definition of a farm changes accordingly.

In summary, from the literature combing in the previous section, it can be seen that domestic and foreign scholars on rural tourism and leisure agriculture concept have been quite a lot of discernment and related research and have also achieved a lot of meaningful results. Therefore, it is necessary for us to make a clear analysis of the concepts of rural tourism and leisure agriculture. Rural tourism and leisure agriculture are different in academic concepts. There is a difference between rural tourism and leisure agriculture, and the concept of rural tourism is larger than leisure agriculture in connotation and extension. Leisure agriculture's central word is agriculture, and leisure exists as a qualifier of agriculture, playing a modifying role.

## 4. Research Methods

ESDA is a combination of statistical principles and visualization techniques such as maps, graphs, and charts to identify and analyze the nature of spatial data without imposing any a priori theoretical or hypothetical premises on the data, and to formulate hypotheses in an inductive manner. The ESDA method builds on the concept of spatial autocorrelation of the first theorem of geography to discover patterns of spatial outliers or spatial agglomerations and reflects the correlation and the degree of correlation of each region through statistics such as Moran's *I* and Geary's C.

### 4.1. Selection of Spatial Weight Matrix

In the spatial analysis, the spatial weight matrix is selected, and since there are many kinds of weight matrices, and the rook spatial weight matrix is the most commonly used, the rook weight matrix of the first order is selected in this paper. Rook first order weight matrix *W* is defined as follows:

(1) $$\begin{array}{c} W_{ij}=\left\{\begin{array}{c} 1\text{ When region }i\text{ region}j\text{ is adjacent,}\\ 2\text{ When region }i\text{ region}j\text{ is not adjacent,} \end{array}\right. \end{array}$$

where *i*=1,2,…, *n*;  *j*=1,2,…, *m*;  *m*=*n* or*m* ≠ *n*.

The article "Econometric Analysis of Leisure Agriculture and Rural Tourism Scenery Based on Spatial Data Analysis" was retracted in 2023. Reasons: unreliable results or conclusions; concerns about the data; concerns about the peer review; concerns about the citations.

### 4.2. Spatial Autocorrelation Analysis

The first law of geography makes the basic assumption of classical statistics about the independence of measurements from each other no longer valid, thus making spatial dependence or called spatial correlation a norm. Spatial statistical analysis Moran's *I* is a statistical analysis technique for analyzing phenomena with spatial dependence.

Moran's *I* is defined as follows:

(2) $$\begin{array}{c} {\text{Moran}}^{\prime }sI=\frac{\sum_{i=1}^{n}\sum_{j=1}^{n}W_{ij}\left(Y_{i}-\bar{Y}\right)\left(Y_{j}-\bar{Y}\right)}{S^{2}\sum_{i=1}^{n}\sum_{j=1}^{n}W_{ij}}, \end{array}$$

where $S^{2}=1/n\sum_{i=1}^{n}{\left(Y_{i}-\bar{Y}\right)}^{2},\;\bar{Y}=1/n\sum_{i=1}^{n}Y_{i}$ is the observed value of the *i*-th region.

If the regions are spatially positively correlated, the value of *I* should be larger; if they are negatively correlated, the value is smaller. When the target region data are similar in spatial location and have similar attribute values, the spatial model as a whole shows positive spatial correlation; while when the spatially neighboring target region data unusually have dissimilar attribute values, it presents negative spatial correlation; when the regional data have zero similar attribute values in spatial location, the spatial model as a whole appears to be independent of each other.

### 4.3. Spatial Econometric Models and Estimation

There are various spatial econometric models. Depending on how the model is set up to reflect the “spatial dependence,” there are two main types of spatial econometric models.

(1) Spatial Lag Model (SLM), which mainly explores whether there is a diffusion phenomenon (spillover effect) of each variable in a region, and its expression is
  (3) $$\begin{array}{c} y=\rho W_{y}+X\beta +\varepsilon . \end{array}$$
(2) Spatial Error Model (SEM), which is used to explain the differences in the interactions between regions due to their relative positions. Its expression is
  (4) $$\begin{array}{c} y=X\beta +\varepsilon ;\varepsilon =\lambda W_{\varepsilon }+\mu . \end{array}$$

## 5. Empirical Analysis

### 5.1. Exploratory Spatial Data Analysis

To describe the spatial distribution of provincial tourism income in China, 31 provinces in mainland China were first used as spatial observation units to conduct spatial autocorrelation tests, which were used to determine whether there was spatial aggregation of tourism income (Figure 1).

The article "Econometric Analysis of Leisure Agriculture and Rural Tourism Scenery Based on Spatial Data Analysis" was retracted in 2023. Reasons: unreliable results or conclusions; concerns about the data; concerns about the peer review; concerns about the citations.

The spatial autocorrelation test (see Figure 1) found that the spatial Moran indices of total tourism income, agricultural and rural tourism income, and agricultural and rural tourism foreign exchange income were 0.4127, 0.4108, and 0.3834, respectively, all of which passed the 1% significance level test. This shows that there is a significant spatial aggregation behavior in the spatial distribution of the explanatory variables TR, DR, and FR. Although the spatial autocorrelation test supports the judgment of spatial dependence, it is not possible to know from the figure which specific provinces belong to which type, and Table 1 is further supplemented in order to more clearly identify each region and its relationship with neighboring regions [21, 22].

As can be seen from Table 1, the regional breakdown of total tourism revenue and agricultural and rural tourism revenue is identical, while the breakdown of foreign exchange earnings from agricultural and rural tourism changes slightly, indicating that agricultural and rural tourism accounts for a very large share of total tourism revenue, while inbound tourism revenue has little impact on total tourism revenue. As can be seen in Figure 1, in 2019, 21 provincial areas of overall tourism and agricultural and rural tourism show similar spatial associations, of which 14 are in quadrant I and 7 in quadrant III; 10 provincial areas show spatial associations with nonsimilar values, of which 6 are in quadrant II and 4 in quadrant IV; 18 provincial areas of agricultural and rural tourism show similar spatial associations. Eighteen provinces showed similar spatial associations for agricultural and rural tourism, 12 of which were in quadrant I and 6 in quadrant III, while 13 provinces showed spatial associations with nonsimilar values, and 7 of which were in quadrant II and 6 in quadrant IV.

### 5.2. Analysis of Tourism Influencing Factors

The spatial dependence of tourism revenues shows that tourism regions do not exist in isolation but are closely related to adjacent or neighboring regions in space, with strong inter-regional influences. Therefore, the spatial effects have to be considered when discussing the factors influencing tourism income. Before spatial econometric estimation, the spatial factor is not considered, but an ordinary least squares estimation of the model is used to compare the analysis with the parameters estimated by the spatial econometric model (Table 2).

As can be seen from Table 2, all three models pass the 1% significance level test. In the total income model and the domestic income model, the level of economic development, tourism enterprises, students, and postal and telecommunications industries all pass the 1% or 5% significance level test, while the foreign openness does not pass the 10% significance level test. In the model of foreign exchange income from agricultural and rural tourism, only the variable of economic development level passed the test of 10% level of significance, while all other variables were not significant, and the OLS estimation of the classical linear regression model may have inappropriate model setting which ignores the spatial effect. In order to further make the problem of the existence of spatial lag model and the choice of spatial error model for the three types of tourism, further judgment is needed [23–25].

The article "Econometric Analysis of Leisure Agriculture and Rural Tourism Scenery Based on Spatial Data Analysis" was retracted in 2023. Reasons: unreliable results or conclusions; concerns about the data; concerns about the peer review; concerns about the citations.

From the results in Table 3, total tourism revenue and domestic revenue LM-lag and Robust LM-lag are highly significant, while LM-error and Robust LM-error do not pass the significance test; therefore, it is judged that a spatial lag model should be selected; foreign exchange revenue both fail the test and fail to build a spatial econometric model. Since the OLS model omits the spatial autocorrelation problem, it leads to the estimated results may not be reliable enough. The SLM model takes into account the spatial effects, so the estimated results are more robust. The following analysis is based on the results of the SLM. For comparison, the results of the SLM are also presented in the foreign exchange earnings model (Table 4).

As can be seen in Table 4, the *ρ*, economic development level, tourism enterprises, and students variables in the total tourism income model and the agricultural and rural tourism income model pass the 1% significance level, while the post and telecommunications industry variable passes the 5% significance level. Combined with the OLS results, the *R*^2^ and the maximum likelihood values are also larger than those estimated by the OLS, while the model has no heteroskedasticity, indicating that the results of these two spatially lagged models are good. On the other hand, the model of foreign exchange earnings from agricultural and rural tourism has serious heteroskedasticity and therefore cannot be spatially modeled.

The error parameters *ρ* of the spatial lag models are 0.1341 and 0.1391 for total tourism revenue and agricultural and rural tourism revenue, respectively, which are significantly positive and both pass the 5% test. This indicates that there is a significant spatial spillover effect of the overall development of tourism and agricultural and rural tourism development in the neighboring provinces to the overall tourism and agricultural and rural tourism development in the region, and this spillover effect of agricultural and rural tourism is greater than that of the overall tourism.

The article "Econometric Analysis of Leisure Agriculture and Rural Tourism Scenery Based on Spatial Data Analysis" was retracted in 2023. Reasons: unreliable results or conclusions; concerns about the data; concerns about the peer review; concerns about the citations.

The level of economic development is the most important factor affecting total tourism income and agricultural and rural tourism income, with each 1% increase in GDP per capita leading to 0.61% increase in total tourism income and 0.62% increase in agricultural and rural tourism income. This indicates that the development of agricultural and rural tourism in China occupies an important position in the overall development of tourism, while the great improvement in the standard of living of Chinese residents will lead to a greater preference for travel. From the previous golden weeks such as the Spring Festival, May Day, and National Day, the tourist attractions are full of tourists, which also fully demonstrates the residents' love and preference for tourism. In this regard, it can be judged that, with the continuous improvement of China's economic development, the demand for tourism will become larger and larger. How to fully meet their growing demand for tourism while providing more tourism services while ensuring the quality of tourism has become a difficult problem in front of scholars and policy makers.

### 5.3. Spatial Econometric Estimation and Analysis of Results

As shown in Table 5 in the results of the spatial error model, the coefficient of the transportation variable measured 31001, which is positive, indicating that the spatial error model has a reasonable probability. Compared to the classical regression, Log likelihood increased from −497.303 to −488.179, AIC decreased from 1008.597 to 991.289, and SC decreased from 1019.651 to 990.239, indicating that the spatial error model has a better fit than the classical regression. The likelihood ratio test LRT = 2.931 with a *p* value of 0.088, the *Z*-value of the spatial autoregressive error coefficient is −2.263, Wald test = (−2.263)^2^  = 5.12, and LM_error = 2.204, which is in line with the expectation of *W* > LRT > LM error, so the spatial error model is judged to be reasonable. Moreover, the significance level of all variables is within 10%, and the spatial autoregressive coefficient is −0.60952, indicating that the correlation effect of its space can be well shown under the condition of spatial error model, and the spatial error model is a relatively good model.

In the spatial error model, the coefficients of the variables in descending order are as follows: service quality > hotel > openness > scenic area > economic level GDP > transportation, that is, the factors affecting foreign tourists agricultural and rural tourism, in order of importance: service quality, hotel, openness, scenic area, economic level, and transportation. This finding differs greatly from the local tourism characteristics of domestic tourists, for domestic tourists, the influence of these six factors may be in order of scenic spots, transportation, hotels, quality of service, economic level, openness, or scenic spots, transportation, quality of service, hotels, economic level, openness quality, and quantity of scenic spots is the most direct factor driving tourist tourism, never put the transportation element at the end. This difference is caused by the unfamiliarity of foreign tourism and the characteristics of Chinese tourism conditions.

The article "Econometric Analysis of Leisure Agriculture and Rural Tourism Scenery Based on Spatial Data Analysis" was retracted in 2023. Reasons: unreliable results or conclusions; concerns about the data; concerns about the peer review; concerns about the citations.

## 6. Conclusion

In this paper, the spatial distribution patterns of agricultural and rural tourism were depicted by using cross-sectional data of agricultural and rural tourism trips, using global and local scatter diagrams and LISA clustering diagrams; the effects of various tourism influencing factors on agricultural and rural tourism were measured by using the classical regression model, SLM, and SEM, respectively. The following conclusions were obtained: (1) agricultural and rural tourism has obvious spatial effects, and the whole area shows positive correlation, and the overall trend is increasing year by year, and the spatial aggregation is becoming more and more obvious; (2) the spatial correlation on the local area varies greatly, with the high-high area in the east and the low-low area distributed in the west, respectively, and the positive region-wide spatial correlation is due to the fact that the low-low area is more than the high-high area, and as the positive global spatial correlation is due to more low-low areas than high-high areas, and the positive low-low correlation on the local area becomes more and more obvious as the year increases. Based on economic growth theory, multiplier theory, and tourism economic effect theory, this paper researches the impact of rural tourism on the regional economy of Chengdu, adds to a certain extent to the research methodology of rural tourism, enriches the research theory in this field, and puts forward relevant countermeasure suggestions, which will provide theoretical guidance and decision-making reference for relevant departments on how to better exert the economic effect of tourism and will also have a certain realistic reference role on how to develop rural tourism in western cities of China.

## Figures and Tables

**Figure 1:** Moran scatter plots of total revenue, domestic revenue, and foreign revenue (logarithmic value).

**Table 1:** Geographic classification in line with Moran scatter plot.

Type	Total tourism revenue	Domestic tourism revenue	Foreign exchange earnings from inbound tourism
High-high	Beijing, Shanxi, Tianjin, Shandong, Henan, Anhui, Hubei	Beijing, Shanxi, Tianjin, Shandong, Henan, Anhui, Hubei, Hunan, Guizhou, Fujian, Guangdong, Jiangsu, Shanghai, Zhejiang	Anhui, Hubei, Hunan, Fujian, Guangdong, Guangxi, Jiangsu, Shanghai, Zhejiang

Low-high	Jilin, Jiangxi, Chongqing, Guangxi, Hebei, Hainan	Jilin, Jiangxi, Chongqing, Guangxi, Hebei, Hainan	Jilin, Shanxi, Henan, Jiangxi, Guizhou, Hebei, Hainan

Low-low	Heilong	Heilong	Xinjiang

High-low	Shaanxi, Yunnan, Sichuan, Liaoning	Shaanxi, Yunnan, Sichuan, Liaoning	Heilongjiang, Inner Mongolia, Shaanxi, Yunnan, Chongqing, Liaoning

The article "Econometric Analysis of Leisure Agriculture and Rural Tourism Scenery Based on Spatial Data Analysis" was retracted in 2023. Reasons: unreliable results or conclusions; concerns about the data; concerns about the peer review; concerns about the citations.

**Table 2:** Results of OLS regressive estimation.

Variable	Total tourism revenue			Domestic tourism revenue			Foreign exchange earnings from inbound tourism		
	Factor	Standard error	Probability	Factor	Standard error	Probability	Factor	Standard error	Probability
Constants	−11.898	3.4258	0.0021	−12.212	3.459	0.0017	−10.559	8.5569	0.2296
AV GDP	0.7258	0.2551	0.0048	0.7432	0.2461	0.0045	1.0399	0.594	0.0887
TE	0.3006	0.1329	0.0329	0.3039	0.1421	0.0336	0.3521	0.3332	0.3079
STU	0.2982	0.0992	0.0039	0.3002	0.0932	0.0023	0.3226	0.229	0.1423
PT	0.5525	0.1712	0.0030	0.5525	0.1695	0.0023	0.4621	0.4221	0.2915
OP	−0.1732	0.1352	0.1928	−0.2219	0.1311	0.1025	0.2988	0.3235	0.3725
Adj *R*^2^	0.902			0.899			0.7501		
Pro (F-statistic)	0.0001			0.0001			0.0001		
Log likelihood	−0.8556			−8.9628			−37.0355		

**Table 3:** Diagnostic for spatial dependence.

Inspection	Total tourism revenue		Domestic tourism revenue		Foreign exchange earnings from inbound tourism	
	Numerical value	Probability	Numerical value	Probability	Numerical value	Probability
LM-lag	6.5225	0.0112	6.6622	0.0097	0.1620	0.6885
Robust LM (lag)	6.9912	0.0085	7.2514	0.0079	0.0869	0.7825
LM-error	0.0325	08525	0.0347	0.8725	0.1529	0.6968
Robust LM (error)	0.5226	0.4789	0.5220	0.4768	0.0795	0.7788

**Table 4:** Results of spatial lag model via maximum likelihood.

Variable	Total tourism revenue			Domestic tourism revenue			Foreign exchange earnings from inbound tourism		
	Factor	Standard error	Probability	Factor	Standard error	Probability	Factor	Standard error	Probability
*ρ*	0.1314	0.0446	0.0041	0.1389	0.0481	0.0034	0.0327	0.0871	0.6912
*C*	−11.787	2.7210	0.0001	−12.041	2.7412	0.0001	−10.558	7.6849	0.1638
AVGDP	0.6213	0.1892	0.0013	0.6213	0.1912	0.0013	1.0088	0.5345	0.0612
TE	0.3981	0.1203	0.0006	0.3981	0.1231	0.0049	0.3806	0.3115	0.2221
STU	0.0701	0.0001	0.3515	0.0752	0.0001	0.3702	0.2219	0.0841	0.1239
PT	0.3386	0.1536	0.0271	0.3241	0.1558	0.0345	0.3672	0.3919	0.4321
OP	−0.1362	0.1021	0.2113	0.1032	0.1063	0.3039	0.3041	0.2658	0.2855
0.20 *R*^2^	0.9267			0.9347			0.7869		
Log likelihood	−4.8302			−5.1721			−37.001		
Breusch–pagan test	2.7188			2.5125			12.6129		

The article "Econometric Analysis of Leisure Agriculture and Rural Tourism Scenery Based on Spatial Data Analysis" was retracted in 2023. Reasons: unreliable results or conclusions; concerns about the data; concerns about the peer review; concerns about the citations.

**Table 5:** Results and diagnostic tests of spatial measures and classical regressions of agricultural and rural tourism in 2012.

Variable	OLS regression		Spatial lag model		Spatial error model	
	Coefficient	*p* value	Coefficient	*p* value	Coefficient	*p* value
*C*	−7602356	0.213	−7715816	0.671	−6254321	0.091
Scen	431211	0.092	426691	0.129	384599	0.023
Hote	842462	0.034	866881	0.047	909881	0.019
Tran	−184771	0.579	−198113	0.009	31115	0.987
Open	851752	0.001	855429	0.497	839651	0.001
Serv	854349	0.687	874252	0.001	1691234	0.035
GDP	1545829	0.001	1487866	0.621	287315	0.001
*ρ* or *λ*	—	—	0.0389	0.001	−0.60887	0.022
*R* ^2^	0.859	—	0.9239	—	0.945	—
Log likelihood	−497.236	—	−491.449	—	−488.179	—
AIC	1008.597	—	995.101	—	991.289	—
SC	1019.651	—	996.102	—	990.239	—
LRT	—	—	0.194	0.669	2.931	0.088
Regression diagnostics			MI/DF	Value	*p* value	
Multicollinearity condition number			—	58.989	—	
Jarque–Bera			3	1.233	0.515	
White			26	27.112	0.476	
Moran's *I*			0.155	—	—	
Lagrange multiplier(lag)			1	0.197	0.655	
Robust LM (lag)			1	0.876	0.355	
Lagrange multiplier (error)			1	2.204	0.097	
Robust LM (error)			1	2.403	0.119	

## Data Availability

The data used in this paper are available from the corresponding author upon request.
